# Stroke and Pneumonia: Mechanisms, Risk Factors, Management, and Prevention

**DOI:** 10.7759/cureus.19912

**Published:** 2021-11-26

**Authors:** Idan Grossmann, Kevin Rodriguez, Mridul Soni, Pranay K Joshi, Saawan C Patel, Devarashetty Shreya, Diana I Zamora, Gautami S Patel, Ibrahim Sange

**Affiliations:** 1 Research, Medical University of Silesia Faculty of Medical Sciences, Katowice, POL; 2 Research, Universidad Americana (UAM) Facultad de Medicina, Managua, NIC; 3 Research, Shri Lal Bahadur Shastri Government Medical College, Mandi, IND; 4 Medicine, Byramjee Jeejeebhoy Medical College, Ahmedabad, IND; 5 Medicine, Pramukhswami Medical College, Karamsad, IND; 6 Internal Medicine, Gandhi Medical College, Secunderabad, IND; 7 General Medicine, Universidad de Ciencias Médicas Andrés Vesalio Guzman, San José, CRI; 8 Internal Medicine, Pramukhswami Medical College, Karamsad, IND; 9 Research, California Institute of Behavioral Neurosciences & Psychology, Fairfield, USA; 10 Research, KJ Somaiya Medical College, Mumbai, IND

**Keywords:** post-stroke pneumonia management, statins and stroke-associated pneumonia, dysphagia and stroke-associated pneumonia, pneumonia prevention in stroke patients, post-stroke pneumonia, stroke-associated pneumonia, pneumonia, stroke

## Abstract

A stroke is a cerebrovascular medical emergency characterized by the sudden loss of neurological function due to interruption to the blood supply. A serious and common complication of stroke is pneumonia. This review article outlined various studies in order to understand the pathogenesis pathways that lead to the development of stroke-associated pneumonia, as well as therapeutic and preventive options to reduce pneumonia. The article looked for risk factors that increase the risk of developing pneumonia among stroke patients. In addition, it has reviewed various therapeutic modalities, such as postural modifications, pharmacological treatment, and other unique treatments, in an attempt to find which of them are efficient to decrease the occurrence of pneumonia and which of them are not. The article also attempts to emphasize the importance of early screening for dysphagia among stroke patients and demonstrates the importance of preventive strategies that can be easily implemented, such as routine oral care and behavioral modifications.

## Introduction and background

Stroke is defined as a cerebrovascular medical emergency characterized by the sudden loss of neurological function attributable to a hemorrhage in the brain tissue or an interruption of the blood supply itself [1].

The term “stroke” was defined in 1599 and was ascribed to an abrupt onset of symptoms that came to be called “apoplexy,” which implied death due to sudden loss of consciousness [2-4]. The prevalence of stroke in elderly patients was 17.8%, while the prevalence in young individuals ranged from 10% to 15%, making it the fifth leading cause of death in the United States [5,6]. According to statistics, 85% of the strokes recorded were known to be ischemic, with a large proportion of them occurring mainly in young individuals of the African population [5-7]. The incidence of stroke depends on the ubiquity of potentially treatable risk factors such as hypertension, hyperlipidemia, diabetes mellitus, and tobacco use [8].

Stroke is a cerebrovascular predicament that is mainly divided into an ischemic stroke, which occurs due to an embolism or in situ small vessel disease, and hemorrhagic stroke, which aspires due to vascular abnormalities such as hypertension or cerebral amyloid angiopathy [9]. Being a repercussion of a medical contingency, stroke tends to present with the abrupt onset of sudden unilateral weakness, numbness, vision loss, diplopia, altered speech, ataxia, and non-orthostatic vertigo with the presence of varying associated symptoms such as headache [9].

The diagnostic modalities indicated in an individual suspected to have a stroke include a contrast computed tomography (CT) or magnetic resonance imaging (MRI) with neuroimaging being used as an essential tool to differentiate between ischemic or hemorrhagic causes and to rule out nonischemic central nervous system abnormalities that might precipitate the condition itself [10,11].

The primary treatment of acute ischemic stroke includes the administration of alteplase within four and a half hours of the onset of symptoms [9]. Mechanical thrombectomy is considered an appropriate management option within 24 hours of the onset of the disease regardless of the alteplase administration for the occurrence of the same ischemic stroke [9]. The pertinent approach to a hemorrhagic stroke includes a gradual reduction in the elevated blood pressure with the cautious use of beta-blockers such as labetalol, calcium channel blockers such as nicardipine, and hydralazine [12]. Considering the essential role played by coagulopathy in the development of stroke, management with agents such as fresh frozen plasma, prothrombin complex concentrate, and factor IX concentrate has been seen to decrease complications and slow the progression of the disease [13]. Pneumonia occurs in 4%-10% of patients experiencing a stroke, making it one of the most problematic complications, associating it with a high mortality rate [14].

Acute stroke gravitates the alteration of peripheral immune responses, resulting in transient lymphopenia and monocyte deactivation, increasing susceptibility to infections [15]. Stroke immunomodulation alters tracheal epithelium, reduces pulmonary clearance, and impairs secretion drainage, which plays a significant role in developing pneumonia [16]. The augmentation of pneumonia is attributed to the presence of risk factors such as stroke severity, loss of consciousness, advanced age, and preexisting comorbidities [17-19].

This review article focuses on evaluating the mechanisms of pneumonia development in stroke patients, exploring the risk factors that increase the likelihood of developing it, and evaluating treatment modalities and preventive strategies to reduce adverse outcomes, curb persistent complications, and improve prognosis over time.

## Review

Stroke-associated pneumonia

Mechanisms

Stroke-associated pneumonia is frequently caused by aspiration. Hospitalized patients suffering from neurological injury have weak swallowing reflexes and are therefore susceptible to developing aspiration [20]. An endotracheal tube is inserted to help protect against large volume aspirations. However, it does not eliminate the possibility of smaller aspirations of pharyngeal or gastric contents. Furthermore, the presence of the endotracheal tube interferes with normal defense mechanisms, such as coughing, and increases the risk of developing ventilator-associated pneumonia [21].

Coughing is an important defense mechanism for protecting against aspirations and the occurrence of pneumonia. Weakening of the cough reflex, as well as impaired swallowing, have been linked to the development of aspiration pneumonia. A prospective study by Nakajoh et al. included 143 consecutive post-stroke patients aged 65 years or older. The combined attenuation of swallowing and cough reflexes appeared to be an important marker for increased pneumonia risk in post-stroke dysphagia patients. The study suggested the use of feeding tube placement in mildly and moderately disabled post-stroke patients with attenuated protective reflexes, who were subjected to increased risk of pneumonia [22].

An observational study conducted by Kulnik et al. in the United Kingdom investigated the effect of cough on the incidence of pneumonia. The study examined it by measuring peak cough ﬂow (PCF) (indicated stronger cough). In this study, 72 patients participated. The participants were adults who were diagnosed with stroke within two weeks, and the study excluded patients with signiﬁcant cardiac/pulmonary disease, neurological conditions other than stroke, orthopedic conditions affecting respiratory mechanics, inability to cooperate, and signs of pneumonia at enrollment. Patients in the low PCF group had a threefold increased risk of pneumonia. The researchers concluded that a strong cough protects against aspiration pneumonia and could be used to predict pneumonia risk in acute stroke patients [23].

Another implicated mechanism in the development of pneumonia after a stroke is attenuated cholinergic pathways. In 2015, Engel et al. carried out an experimental study in Germany using a middle cerebral artery occlusion model in mice to investigate the role of the parasympathetic nervous system in post-stroke immunosuppression. According to the findings, inhibiting cholinergic signaling by vagotomy or using nicotinic acetylcholine receptor-deficient mice stimulated an increased immune response and prevented pneumonia after stroke. Those results showed an association between the cholinergic pathway and the risk of developing pneumonia [24].

Due to decreased mastication, salivation, swallowing, and oral hygiene, patients with acute stroke are especially vulnerable to disruption of the oral microbial ecology. The presence of pathogenic oral bacteria in post-stroke patients is associated with a poor prognosis, which leads to aspiration pneumonia [25].

Risk Factors

Severe hypertension is one of the most important risk factors for developing stroke-associated pneumonia. A comparative study by Ishigami et al. took place in the Geriatric Emergency Ward of Kanazawa Medical University Hospital in Japan. The study included 118 patients diagnosed with ischemic stroke during 2002-2010; the patients were 70 years of age or older and had both clinical and neuroimaging evidence of ischemic cerebral infarction. The finding showed a significant association of severe hypertension, defined as 200/120 mm Hg or higher, on admission with the occurrence of stroke-associated pneumonia [26].

Another Japanese study, which tried to understand the risk factors for developing pneumonia among stroke patients, was conducted by Matsumura et al. in 2014. The study included 76 stroke patients with dysphagia. Of the patients, 13.2% developed pneumonia at the hospital, and all of them were over the age of 65. This study concluded that recumbency, malnutrition, tube feeding, severe dysphagia, and female sex were all risk factors for pneumonia [27].

Immunodeficiency is another factor that has been linked to pneumonia because of aspiration, which is a primary mechanism for developing stroke-associated pneumonia. In a newly developed model of post-stroke pneumonia, Prass et al. conducted an experimental study in 2006 to examine if stroke-induced immunodeficiency increases the risk of pneumonia after aspiration. Mice aged nine to 13 weeks made up the population of this experiment. Immunodepression was discovered to be necessary for the progression of bacterial aspiration to pneumonia [28].

Another retrospective study was conducted between 2000 and 2009 by Sui et al. in China to explore the risk factors in the Chinese population in order to better understand the development of pneumonia in post-stroke patients. Researchers discovered that diabetes, age, consciousness, days in the hospital, tracheal intubation, tracheal incision, nasal feeding treatment, and the use of H2-receptor blocking agents and antimicrobials were all linked to stroke-related pneumonia [29].

Between 2008 and 2013, Bruening et al. conducted a prospective study with 538 participants to examine the link between pneumonia and prognosis in stroke patients receiving intravenous thrombolysis with recombinant tissue plasminogen activator. At the University of Lübeck’s Department of Neurology, 538 consecutive stroke patients were given intravascular (IV) thrombolysis, and the findings revealed that the incidence of stroke-associated pneumonia was linked to increased age, male sex, the severity of neurological deficits, and the length of hospitalization [30].

Stroke-related pneumonia has been linked to a variety of chronic inflammatory diseases. Dylla et al. investigated the link between various chronic inflammatory diseases and the incidence of stroke-related pneumonia. Adults with acute ischemic stroke who were 18 years old were included in this cohort study, which used data from 2015 to 2017 in the United States. The findings suggested a complex interplay between various inflammatory diseases and the likelihood of stroke-related pneumonia. The conclusion was that more research is required to determine the link between those diseases and stroke-related pneumonia. A better understanding of the link could lead to a reduction in stroke-related pneumonia [31].

*Streptococcus mitis*, *Streptococcus pneumoniae*, *Staphylococcus aureus*, *Klebsiella pneumoniae*, *Escherichia coli*, and *Pseudomonas aeruginosa* are six bacteria that have been linked to aspiration pneumonia [32-35]. In order to determine the relationship between oral bacteria and pneumonia in a clinical stroke population, Perry et al. conducted a study in New Zealand that included 102 patients with acute stroke and measured the relative amounts of change in bacteria over time for some species. It was found that the levels of some bacteria were higher in discharge and one month after discharge than it was on admission. The study also demonstrated that the change in bacteria levels is associated with the development of pneumonia. The researchers concluded that the presence of respiratory flora in patients’ mouths within 48 hours of a stroke is clinically significant [36].

Management and Prevention

Pneumonia is a common complication of stroke, and therefore, it requires appropriate diagnostic criteria, as well as strategies for the management and prevention of its development. Currently, there is no agreed-upon terminology or gold standard diagnostic criteria for the spectrum of lower respiratory tract infections that complicate stroke. Smith et al. proposed consensus operational criteria for the diagnosis and management of stroke-associated pneumonia in the United Kingdom in 2014. According to this criteria, stroke-associated pneumonia is diagnosed by progressively infiltrating lesions in post-stroke chest images, as well as more than two of the following clinical symptoms of infection: (1) 38°C fever; (2) newly occurring cough, productive cough, or exacerbation of preexisting respiratory disease symptoms with or without chest pain; (3) signs of pulmonary consolidation and/or moist rales; and (4) peripheral WBC above 10 × 10^9^/L or below 4 × 10^9^/L with or without a nuclear shift to the left. Furthermore, some diseases with similar clinical manifestations to pneumonia, such as tuberculosis, pulmonary tumor, noninfective interstitial lung disease, pulmonary embolism, and pulmonary atelectasis and pulmonary edema, were ruled out [37].

Although stroke-related pneumonia is a common and serious complication, there are not many standardized antibiotic treatment recommendations for this condition. A survey study was conducted in Germany in 2010 and included a standardized questionnaire for the 83 German stroke units that took part in the study. The study showed that in empiric monotherapy (58%) and combination therapy (42%), group 3 cephalosporins and (acyl-)aminopenicillins/beta-lactamase inhibitors were the most commonly used antibiotics (46%-60%). Prophylactic antibiotic treatment was used by a small percentage of stroke units (5%). This study strongly suggested that more research be conducted to establish a standard treatment for pneumonia in stroke patients [38].

Antibiotic prophylaxis does not always work to prevent pneumonia in stroke patients. Between 2008 and 2014, Kalra et al. conducted a prospective study in the United Kingdom to assess the effectiveness of antibiotic prophylaxis in reducing pneumonia in patients with dysphagia after acute stroke. Patients over the age of 18 with dysphagia following a new stroke were recruited from 48 stroke units across the United Kingdom. Patients with antibiotic contraindications, preexisting dysphagia, or known infections were excluded, as were those who were not expected to survive more than 14 days. The study included 1217 people who were divided into two groups: those who were given antibiotics and those who were not. Prophylactic antibiotics did not reduce the incidence of post-stroke pneumonia, and the results did not show a significant difference between the two groups. As a result, antibiotic prophylaxis was not recommended to prevent post-stroke pneumonia in stroke patients [39].

Postural modification may aid in the prevention of aspiration in patients with dysphagia. In 2017, Alghadir et al. conducted a study in Saudi Arabia, where a total of 186 healthy adult males aged 20-40 years old took part in the study. They were evaluated for neurological or musculoskeletal pain and were excluded if any sign or symptom was discovered. The study discovered that in certain positions, it was more difficult to swallow. Different head and neck positions can aid in the swallowing process, allowing to avoid and treat aspirations that could lead to pneumonia. Postural modification may aid in the treatment of dysphagia by improving swallowing speed and preventing aspiration. Reclining position eases the passage of the food because of the gravity. This method is part of the routine of management to prevent aspirations, which is a primary mechanism to develop pneumonia [40].

Systemic oral hygiene care may be one preventive strategy for stroke-associated pneumonia. Between 2008 and 2013, Wagner et al. conducted a cohort study in Boston, Massachusetts, involving 1656 stroke patients. The patients were split into two groups: control and intervention (which received systemic oral hygiene treatment). The rate of stroke-related pneumonia was lower in the intervention group than in the control group. The conclusion was that proper oral hygiene is linked to a lower risk of pneumonia in stroke patients. Thus, a simple routine of oral care among stroke patients can help reduce pneumonia incidence (Table 1, Figure 1) [41].

**Figure 1:** The effect of oral hygiene care on the percentage of pneumonia cases

Dysphagia, as previously mentioned, is a risk factor for stroke-related pneumonia. Early dysphagia screening could help prevent stroke-related pneumonia. Between 2007 and 2012, Al-Khaled et al. conducted a hospital-based study that included 9164 patients with acute ischemic stroke who were residents of the German state of Schleswig-Holstein. Patients who presented to the emergency department but declined hospital admission and those who were admitted with suspected acute ischemic stroke but later received a different diagnosis were excluded from the study. Patients with dysphagia had higher rates of pneumonia than those without dysphagia, and early dysphagia diagnosis within 24 hours of admission appeared to be associated with a lower risk of stroke-related pneumonia. The conclusion was that dysphagia places stroke patients at an increased risk of pneumonia, and early dysphagia screening was associated with a lower risk of stroke-related pneumonia (Table 1) [42]. Another study that supported the important role of dysphagia screening in reducing the number of pneumonia cases in acute ischemic stroke patients was conducted by Yeh et al. The study included patients who were admitted to the intensive care unit in National Taiwan University Hospital between 2006 and 2007. Overall, 176 patients participated in this study. The exclusion criteria were patients who were intubated on the first day of admission and patients who had a transient ischemic attack. Dysphagia screening was associated with a decrease in stroke-associated pneumonia in all stroke patients, and the study concluded that the dysphagia screening could help prevent stroke-associated pneumonia [43].

Beta-blockers may also help reduce the risk of post-stroke pneumonia. Sykora et al. analyzed 5212 patients in a nonrandomized comparison study in Germany in 2015. A total of 1155 (22.2%) patients were treated with beta-blockers prior to the onset of the stroke, and 244 (4.7%) patients were started on beta-blockers during the acute phase of the stroke. Beta-blockers were found to be linked to a lower risk of pneumonia both before and after a stroke. The researchers recommended that more research should be done to see if beta-blockers could be used as part of the treatment for acute stroke [44].

Vitamin E may be beneficial to patients suffering from stroke-related pneumonia. In a prospective study conducted at the Neurology Department of Qingdao Municipal Hospital Group in China by Shen et al. in 2019, 183 patients with stroke-related pneumonia were selected and divided into different nutrition groups. For each group, a different dose of vitamin E was given, and it was discovered that patients in the high-dose vitamin E group had better immune system function and hospitalization than those in the low-dose vitamin E group. The researchers concluded that vitamin E might have a supplementary therapeutic effect in patients suffering from stroke-related pneumonia (Table 1) [45].

Another treatment option is cilostazol, which has been shown to be effective in preventing stroke-related pneumonia. Netsu et al. conducted a retrospective study in which 158 patients were recruited, and all of them were admitted to Tokai University Hospital between 2009 and 2014 due to ischemic stroke. They met the following criteria: in the acute phase, required intensive care unit management, admitted within a week of onset, magnetic resonance imaging revealed an ischemic lesion, and received tube feeding via nasogastric tube within a week of onset. It was discovered that cilostazol significantly reduced the incidence of stroke-related pneumonia [46].

Statins may help in the prevention of pneumonia and improve prognosis. Scheitz et al. conducted a retrospective study in Germany between 2005 and 2010 that included 481 ischemic stroke patients. All of the patients had an acute ischemic stroke and were treated with a tissue plasminogen activator (tPA) within four and a half hours. The findings revealed that patients who took statins had a lower risk of post-stroke pneumonia than those who did not. The researchers concluded that statin use in acute ischemic stroke patients receiving thrombolysis might lower the risk of post-stroke pneumonia. More research is required to confirm this finding [47]. Similarly, another study that enhanced the former looked at the effect of statins on the risk of developing post-stroke pneumonia. A retrospective observational research study conducted by Song et al. in South Korea included 7001 patients discharged with acute ischemic stroke and no prior history of pneumonia. The study found a reduced risk of post-stroke pneumonia with statin therapy after acute ischemic stroke. It suggested that treatment with statins may have a preventive effect against the common complication of post-stroke pneumonia (Table 1) [48].

In general, acid-suppressive medications have been linked to a higher risk of nosocomial pneumonia in hospitalized patients. Herzig et al. in Boston conducted a cohort study that looked into the link between acid-suppressive medication and hospital-acquired pneumonia in patients with acute stroke. Between 2000 and 2010, the study included 1340 patients hospitalized with acute ischemic stroke or intracerebral hemorrhage. Patients had to be over the age of 18 and have been in the hospital for at least two days. The findings showed that those who were given acid-suppressive medication had a higher rate of hospital-acquired pneumonia than those who were not. The findings suggested that these medications should be used more cautiously in stroke patients, particularly those considered to be at high risk of pneumonia [49].

Benzodiazepines have been linked to the development of stroke-related pneumonia. Lin et al. conducted a retrospective cohort study to see if there was any correlation. The research was conducted in Taiwan and included 7516 patients newly diagnosed with stroke between 2000 and 2012. The patients were split into two groups: those who received benzodiazepines and those who did not. Over the course of a month after the stroke, 1027 patients in the benzodiazepine group and 478 patients in the non-benzodiazepine group developed pneumonia, according to the findings. Patients who took benzodiazepines after a stroke had had a higher risk of pneumonia than those who did not. Therefore, those who used benzodiazepines had a higher risk of chronic-onset post-stroke pneumonia, according to the study. Hence, although the cause-effect relationship requires further investigation, the results should be considered in an attempt to prevent pneumonia among stroke patients (Table 1) [50].

Metoclopramide, a dopamine receptor antagonist with antiemetic and gastric prokinetic properties, may help reduce the rate of aspiration and pneumonia. Warusevitane et al. studied the efficacy of metoclopramide in reducing pneumonia between 2008 and 2011 in the United Kingdom. The study included 60 patients who had a computed tomography-confirmed acute ischemic or hemorrhagic stroke and needed nasogastric feeds for more than 24 hours and who could be recruited within 48 hours of nasogastric tube insertion. Signs and symptoms of pneumonia after a stroke, a history of chronic neurodegenerative diseases that could affect swallowing (e.g., Parkinson’s disease and motor neuron disease), esophageal disorders, and metoclopramide contraindications were among the study’s exclusion criteria. The results showed that patients who received metoclopramide had a higher rate of pneumonia than those who did not. According to the results, it was concluded that metoclopramide might reduce the rate of pneumonia and improve other clinical consequences in patients with subacute stroke who are fed through a nasogastric tube [51].

Furthermore, acupuncture is now widely recognized as a treatment option for stroke survivors around the world. The Chang et al. retrospective cohort study in Taiwan, which included patients who had a stroke between 2000 and 2004, aimed to assess the protective effect of pneumonia in stroke patients. The patients were divided into a group who received acupuncture after discharge and another group who did not. The study included 12557 stroke patients, with pneumonia being diagnosed in 6796 of them (27.1%). Stroke patients who received acupuncture had a lower rate of pneumonia than stroke patients who did not receive acupuncture (53.4% versus 58.9%, respectively). Thus, acupuncture-treated stroke patients had a lower risk of pneumonia than those who did not. More randomized control trials are required (Table 1) [52].

Acute stroke patients may benefit from transcutaneous electrical stimulation as a treatment option. In a retrospective study conducted by Hamada et al. in the Stroke Care Unit and Rehabilitation Center of Aizawa Hospital between 2010 and 2011, 53 patients were analyzed and divided into two groups: those who received therapy and those who did not. In the patients who received therapy, the risk of pulmonary infection was significantly reduced. Surface electrical stimulation therapy was found to reduce the occurrence of pulmonary infection in post-stroke patients effectively, but more research is required to accurately estimate the therapy’s effects in this population (Table 1) [53].

**Table 1:** Summary of the included studies on stroke-associated pneumonia prevention strategies

Reference	Design	Number of participants	Population	Conclusion
Wagner et al. (2016) [41]	Cohort study	1656	Hospitalized stroke patients before and after implementation of a systemic oral hygiene care innervation	Proper oral hygiene care is linked with a lower risk of pneumonia in stroke patients
Al-Khaled et al. (2018) [42]	Hospital-based study	9164	Patients with acute ischemic stroke who were residents of the German state of Schleswig-Holstein	Early dysphagia diagnosis within 24 hours of admission appeared to be associated with a lower risk of stroke-related pneumonia
Shen et al. (2020) [45]	Prospective study	183	Patients with stroke-related pneumonia	Vitamin E may have a supplementary therapeutic effect in patients suffering from stroke-related pneumonia
Song et al. (2020) [48]	Retrospective observational study	7001	Patients with acute ischemic stroke and no prior history of pneumonia	Treatment with statins have a preventive effect against post-stroke pneumonia
Lin et al. (2019) [50]	Population-based cohort study	7516	Patients newly diagnosed with stroke between 2000 and 2012	Benzodiazepines have a higher risk of chronic-onset post-stroke pneumonia
Chang et al. (2018) [52]	Retrospective cohort study	12557	New stroke patients who did and did not receive acupuncture post-stroke	Acupuncture-treated stroke patients had a lower risk of pneumonia than those who did not
Hamada et al. (2017) [53]	Retrospective study	53	Acute stroke patients with dysphagia	Surface electrical stimulation may be effective in reducing the occurrence of pulmonary infection in post-stroke patients

Limitations

This review article presented various preventive strategies, but some of the proposed strategies still require additional evaluation and research to improve and confirm their efficacy. Furthermore, because therapeutic care for stroke-related pneumonia was relatively low over the years and evidence-based guidelines are quite limited, it was difficult to outline one favorable therapeutic and preventive strategy, and no strategy was evaluated for superiority over others.

## Conclusions

This review article addresses the problematic association between stroke patients and their risk of developing pneumonia. In order to reduce the morbidity of stroke-associated pneumonia, this article attempts to assess the mechanisms that lead to the development of pneumonia and to look for the appropriate management and preventive strategies. Coughing and swallowing reflexes are the most crucial protective mechanisms to prevent aspiration pneumonia, which are frequently impaired in post-stroke patients, leading to pneumonia. As a result, aspirations can be formed, and it is the primary mechanism for developing stroke-associated pneumonia. Although pneumonia is a common complication, antibiotic prophylaxis is not recommended for the prevention of post-stroke pneumonia. On the other hand, there are other modalities that can help reduce the occurrence of post-stroke pneumonia. Beta-blockers and statins were found to be linked to a lower risk of pneumonia. Other drugs, such as benzodiazepines, are found to be associated with an increased risk of pneumonia. Acid-suppressive medications have been linked to a higher risk of nosocomial pneumonia, and those medications should be carefully used. Furthermore, special methods such as surface electrical stimulation therapy effectively reduced the occurrence of pulmonary infection in post-stroke patients. This article’s clinical significance is to raise the awareness of physicians who care for these patients and introduce them to a variety of therapeutic and preventive modalities that can help reduce the development of pneumonia in stroke patients. Understanding the mechanisms and risk factors, as well as attempting to reduce them, will aid in the prevention of stroke-related pneumonia. The postural modification will assist patients with dysphagia in avoiding aspiration and, as a result, the development of pneumonia. Furthermore, early dysphagia screening is an option that could help prevent stroke-related pneumonia, and an oral care routine may also help in this purpose. Although stroke-associated pneumonia has been a severe complication among these patients, the information and research regarding this topic are limited, and the management is not definitive and conservational in some cases. In addition, some preventive strategies mentioned throughout this article need further studies in order to be confirmed.
